The article "Effects of High-Frequency Chest Wall Oscillation Expectoration System on Pulmonary Rehabilitation and Cortisol Function in Patients with Severe AECOPD" was published in 2022. Journal: Dis Markers.

# Effects of High-Frequency Chest Wall Oscillation Expectoration System on Pulmonary Rehabilitation and Cortisol Function in Patients with Severe AECOPD

**DOI:** 10.1155/2022/3380048

**Published:** 2022-07-22

**Authors:** Guohua Cheng, Jialing Wu, Zizi Hu, Yumie Xiao, Biyuan Zeng, Yuqiong Zhou

**Affiliations:** Rehabilitation Department, Fourth Hospital of Changsha, Changsha 410005, China

## Abstract

**Objective:**

To investigate the effect of high-frequency chest wall oscillatory expectoration system (HFCWO) on pulmonary rehabilitation and cortisol function in patients with severe acute exacerbation of chronic obstructive pulmonary disease (AECOPD).

**Methods:**

The 65 severe AECOPD patients admitted to our hospital from January 2019 to May 2020 were divided into group A with 33 cases and group B with 32 cases by random number table method. After 14 days of intervention, the improvement time of clinical symptoms in the two groups was recorded, and blood gas, lung function, inflammatory, and cortisol function-related indicators were evaluated before and after treatment.

**Results:**

The remission time of expectoration, pulmonary signs, and hospital stay in group A were significantly shorter than those in group B (*P* < 0.05). Compared with before treatment, blood oxygen partial pressure (PaO_2_), forced vital capacity (FVC), forced expiratory volume at 1 s (EFV1), and EFV1/FVC increased significantly; blood carbon dioxide partial pressure (PaCO_2_), C-reactive protein (CRP), interleukin-6 (IL-6), white blood cell count (WBC), plasma cortisol (COR), and adrenocorticotropic hormone (ACTH) levels were significantly decreased, and the above indicators in group A increased or decreased more significantly than those in group B (*P* < 0.05); there was no significant difference in tolerance and adverse reactions between the two groups (*P* > 0.05).

**Conclusion:**

HFCWO has good pulmonary rehabilitation effect in the treatment of severe AECOPD and can significantly improve the blood gas indexes, inflammation, and cortisol function of patients, which is safe and feasible.

## 1. Introduction

The chronic obstructive pulmonary disease (COPD) is manifested as symptoms of cough and asthma, etc., mainly due to airflow obstruction, and manifested as markedly abnormal lung function during acute exacerbations, which can be life-threatening in severe cases [1]. According to relevant reports, the mortality of the acute exacerbation of chronic obstructive pulmonary disease (AECOPD) is predicted to be among the top five worldwide, and the cause of death is associated with excessive phlegm and ineffective drainage [2, 3]. Therefore, pulmonary rehabilitation is crucial for patients with AECOPD, and physical therapies are the most widely used to improve respiratory symptoms and lung volumes and to shorten recovery time [4, 5]. As two commonly used pulmonary physiotherapies, both high-frequency chest wall oscillation (HFCWO) and expiration with the glottis open in the lateral posture (ELTGOL) can effectively improve the lung function and blood gas indicators of patients with AECOPD, and HFCWO is better as shown by some studies [6], but there are relatively few relevant reports in China. In addition, it was found that the abnormally increased plasma cortisol (COR) in patients with AECOPD is likely to cause adrenocortical dysfunction or aggravate the disease [7]; and adrenocortical function may be related to many factors such as inflammation and low oxygen [8]. In this regard, this study not only analyzed the effect of HFCWO on the pulmonary rehabilitation of patients with severe AECOPD from clinical symptoms, pulmonary function, and blood gas indicators but also explored its feasibility from COR and inflammatory indicators, to provide a reference for the further application of HFCWO in clinical practice. The report is as follows.

## 2. Materials and Methods

### 2.1. Patient Information

Sixty-five patients with severe AECOPD, who were admitted to our hospital from January 2019 to May 2020, were used as subjects and divided into group A (33 cases) and group B (32 cases) using the table of random numbers. Group A consisted of 23 males and 10 females, with an age of 60-85 years, averaged at 67.36 ± 5.95, with COPD duration of 5-40 years, averaged at 11.67 ± 4.52 years, including 12 cases complicated with diabetes mellitus and 15 cases complicated with hypertension. Group B consisted of 21 males and 11 females, with an age of 63-89 years, averaged at 68.03 ± 4.76, with COPD duration of 7-35 years, averaged at 12.34 ± 3.06 years, including 13 cases complicated with diabetes mellitus and 13 cases complicated with hypertension. The baseline data of the two groups were matched (*P* > 0.05) and comparable. The study was approved by the ethics committee of the hospital.

### 2.2. Inclusion and Exclusion Criteria

Inclusion criteria were as follows: (1) consistent with AECOPD-related criteria [9], confirmed by clinical and imaging diagnosis; (2) age > 18 years; (3) clear consciousness and normal reading and writing; (4) able to cooperate with the treatment and examination of this study; (5) no more than 10 d of acute exacerbation; and (6) informed and signed the consent form.

Exclusion criteria were as follows: (1) organic lesions; (2) fractures; (3) large amounts of pus visible in the chest; (4) presence of primary suprarenal lesions or other endocrine symptoms; (5) confusing symptoms such as pulmonary embolism and bronchiectasis; and (6) malignancy, blood coagulation disorders, and dysimmunity.

### 2.3. Methods

Patients in the 2 groups received routine comprehensive treatment according to the *Chinese Expert Consensus on the Diagnosis and Treatment of AECOPD* (updated version in 2017) [9], such as oxygen therapy, respiratory support, relieving cough and asthma, anti-infection, or nutritional support. In addition, HFCWO intervention was given to group A: select the supine position or lateral position as the case may be, clear the airway, put the towel on the back and the forebreast, set the frequency to 10-12 Hz, pressure to about 5 kPa, and time to 15-20 min, and press the start button to start vibration after the above preparation is completed. The secretions during treatment, if any, were promptly aspirated and removed. After the treatment, secondary cleaning was performed to the patient's respiratory tract. ELTGOL was performed to patients in group B: select the lateral position, let the patient breathe normally, open the glottis through the throat and tongue when the residual volume is reached slowly to ease the airway compression, and press the abdomen when the patient slowly exhales, which is similar to the left chest wall compression in principle and was aimed at promoting air escape. The procedure was about 5 min a time, repeated once every 2 min, and repeated 3 times. The patient maintained the right lateral posture during rest. The 14 d intervention was performed for both groups. The therapeutic schedule was timely adjusted in case that the patient's condition worsened or the effects were not obvious.

### 2.4. Observational Indicators

#### 2.4.1. Improvement of Symptoms

The remission time of expectoration and pulmonary signs and the length of stay (LOS) were recorded for patients in the 2 groups.

#### 2.4.2. Blood Gas Indicators

The partial pressure of oxygen (PaO_2_) and the partial pressure of carbon dioxide (PaCO_2_) of the 2 groups were determined by the automatic blood gas analyzer.

#### 2.4.3. Pulmonary Function

The forced vital capacity (FVC) and the forced expiratory volume in the first second (FEV1) of the 2 groups were measured by the pulmonary function tester, and FEV1/FVC was calculated.

#### 2.4.4. Inflammatory Indicators

Fasting blood was collected in the morning. C-reactive protein (CRP) and interleukin-6 (IL-6) of the 2 groups were determined by the enzyme-linked immunosorbent assay (ELISA), and blood routine examination was performed to obtain the white blood cell count (WBC).

#### 2.4.5. Cortisol Function

Fasting blood was collected in the morning. The plasma COR and adrenocorticotrophic hormone (ACTH) of the 2 groups were measured by chemiluminescence.

The above indicators were measured before treatment and after 14 d of treatment. In addition, the tolerance and adverse reactions during treatment were observed for the 2 groups.

### 2.5. Statistical Processing

SPSS 20.0 statistical software was used to process the data. Enumeration data were expressed as cases (%). Measurement data following the normal distribution were expressed as $\bar{x}\pm s$. The *t* test, with the size of test *α* = 0.05, was adopted.

## 3. Results

### 3.1. Improvement of Symptoms

The remission time of expectoration and pulmonary signs and the length of stay (LOS) of patients in group A were significantly shorter than those of group B (*P* < 0.05). See Table 1.

### 3.2. Blood Gas Indicators

After treatment, significantly increased PaO_2_ and significantly decreased PaCO_2_ were observed for both groups. Moreover, after treatment, group A had significantly higher PaO_2_ and lower PaCO_2_ than group B. The differences were statistically significant (*P* < 0.05). See Table 2.

### 3.3. Pulmonary Function

After treatment, FVC, FEV1, and FEV1/FVC obviously increased in both groups and were significantly higher in group A than in group B (*P* < 0.05). See Table 3.

### 3.4. Inflammatory Indicators

WBC, CRP, and IL-6 decreased significantly in both groups after treatment compared with those before treatment and were significantly lower in group A than in group B after treatment (*P* < 0.05). See Table 4.

### 3.5. Cortisol Function

COR and ACTH decreased significantly in both groups after treatment compared with those before treatment and were significantly lower in group A than in group B after treatment (*P* < 0.05). See Table 5.

### 3.6. Safety Evaluation

In group A, 31 cases (93.94%) did not have any discomfort, and 2 cases (6.06%) experienced mild accelerated heart rhythm during treatment. In group B, 28 cases (87.50%) tolerated the treatment without any discomfort, and 4 cases received intermittent treatment due to unskillfulness but did not have any adverse reactions. There was no significant difference in tolerance and adverse reactions between the 2 groups (*P* > 0.05).

## 4. Discussion

It is reported that AECOPD is an important factor leading to reduced lung function and death of patients [10]. Most patients with AECOPD receive comprehensive treatment of oxygen inhalation, eliminating phlegm and anti-inflammation, which can effectively improve symptoms including cough and restore the patient's breathing. However, conventional interventions generally have long cycles and poor clinical outcomes [11–13].

In recent years, physical therapy, such as common means of HFCWO and ELTGOL, has been frequently used for treating AECOPD [14, 15]. Our study shows that shorter remission time of expectoration and lung signs and much more obvious improvement of blood gas indicators and lung function can be observed in patients treated by HFCWO in comparison with those treated by ELTGOL. The reason for this is as follows: with respect to HFCWO, the patient's chest wall is slowly compressed and released through inflation and deflation. The generated airflow in the lungs drives the sputum to the large airway, and the mucus is eliminated with the help of coughing or inspiration [16]. It can evenly act on the patient's chest wall, change the nature of secretions through the mechanics principle, debond secretions in the terminal bronchus, and drive them to the large airway in the middle [17, 18]. HFCWO can significantly improve the efficiency of sputum drainage, increase the effectiveness of atomization intervention, and better improve the clinical symptoms of patients with AECOPD [19]. Meanwhile, the system has biofeedback and other related configurations, which is conducive to enhancing the sputum excretion ability of the body and reducing the number of coughs. Moreover, the system determines lung resonance frequency and viscosity, etc., calculates the strongest resonance, promotes the excretion of mucous secretions as much as possible, and can maximize sputum excretion more comprehensively and objectively compared to ELTGOL. It is reported in the literature that patients with moderate to severe COPD had significantly decreased sputum excretion and significantly improved dyspnea after HFCWO intervention [20]. Chakravorty et al. [21] also found that HFCWO had apparent advantages in improving pulmonary function of patients with COPD and reducing the risk of acute exacerbations. The findings of the present study are consistent with the above, reconfirming the therapeutic value of HFCWO in patients with severe AECOPD.

AECOPD has a complex pathogenesis, mostly involving viral or bacterial infections [22]. Increased serum levels of WBCs and interleukins suggest the presence of lower airway bacterial colonization, and abnormal inflammatory factors aggravate the disease [23]. CRP, WBC, and IL-6 are common inflammatory indicators. The above indicators are frequently used to assess the AECOPD condition, but the specificity is relatively poor. Recently, some scholars point out that AECOPD is associated with inflammation and hormonal imbalance, which lead to persistent damage to the patient's airway, consequently aggravating the disease [24]. COR is closely related to the body's stress response and plays a certain role in the body's environmental balance and stabilization and blood pressure regulation [25]. In addition, COR content is related to the hypothalamic-pituitary-adrenal axis, belonging to glucocorticoids; ACTH, however, can regulate hormones and is positively correlated with the COR content [26]. Reduced lung function, more sputum, and strong inflammation in patients with AECOPD aggravate lung injury and involve the kidney, resulting in reduced renal output and slower COR degradation. In addition, the progression of the disease affects the suprarenal function, further affecting COR decomposition, but its secretion and synthesis increase. The imbalance leads to the increase of serum COR level of the patient [27]. Our study showed that serum inflammatory indicators and plasma COR and ACTH levels decreased significantly after 14 d of HFCWO and ELTGOL treatment and that the relative decrease of the former was more remarkable, suggesting that both HFCWO and ELTGOL can effectively reduce the inflammatory reaction and improve cortisol function in patients with AECOPD. Promoting lung deflation by opening the glottis, ELTGOL can effectively eliminate the airway inflammation of patients, relieve dyspnea, and suppress the disease [28]. However, HFCWO has an advantage over ELTGOL in reducing inflammatory reaction and regulating cortisol function. Retention of more viscous airway secretions in patients with AECOPD can result in bacterial reproduction and aggravate lung infection. With the above advantages, HFCWO can realize more complete sputum removal compared with ELTGOL. The cortisol function of patients with COPD is influenced by many factors such as inflammation and hormones [29, 30]. The impact of different physical therapies on cortisol function of AECOPD patients shall be further confirmed by large sample and multicenter studies in the future. In addition, good tolerance without any obvious adverse reaction was observed for both groups. However, contraindications of HFCWO, such as bleeding, pulmonary embolism, fracture, or empyema, shall be noted in the actual use. The clinical indications and contraindications should be strictly controlled.

In conclusion, compared with ELTGOL, HFCWO shows more evident improvement on clinical symptoms, blood gas, pulmonary function, and cortisol function-related indicators in patients with severe AECOPD, which can be further studied and applied.

## Figures and Tables

**Table 1:** Comparison of symptom improvement between the two groups ($\bar{x}\pm s$, d).

Group	Sputum relief time	Remission time of lung signs	The length of time
Group A (*n* = 33)	3.45 ± 1.20	4.42 ± 1.00	10.61 ± 2.50
Group B (*n* = 32)	4.34 ± 0.97	5.94 ± 1.61	15.56 ± 3.26
*t*	-3.276	-4.576	-6.889
*P*	0.002	<0.001	<0.001

**Table 2:** Comparison of blood gas indexes between the two groups ($\bar{x}\pm s$, mmHg).

Group	PaO_2_		PaCO_2_	
	Before the treatment	After treatment	Before the treatment	After treatment
Group A (*n* = 33)	71.06 ± 9.85	89.30 ± 8.52^∗^	61.85 ± 6.66	44.06 ± 5.81^∗^
Group B (*n* = 32)	70.75 ± 10.70	82.94 ± 7.82^∗^	61.56 ± 7.68	48.06 ± 5.98^∗^
*t*	0.122	3.137	0.161	-2.735
*P*	0.903	0.003	0.873	0.008

Note: vs. before treatment, ^∗^*P* < 0.05; PaO_2_: partial pressure of blood oxygen; PaCO_2_: partial pressure of carbon dioxide.

**Table 3:** Comparison of pulmonary function changes between the two groups ($\bar{x}\pm s$, %).

Group	FVC		EFV1		EFV1/FVC	
	Before the treatment	After treatment	Before the treatment	After treatment	Before the treatment	After treatment
Group A (*n* = 33)	55.24 ± 6.93	64.55 ± 6.72^∗^	37.88 ± 8.43	48.03 ± 7.04^∗^	54.36 ± 4.71	87.36 ± 10.96^∗^
Group B (*n* = 32)	55.25 ± 6.62	60.41 ± 5.99^∗^	38.19 ± 6.58	43.81 ± 6.28^∗^	55.28 ± 4.95	80.47 ± 7.86^∗^
*t*	-0.005	2.618	-0.164	2.547	-0.766	2.907
*P*	0.996	0.011	0.870	0.013	0.446	0.005

Note: vs. before treatment, ^∗^*P* < 0.05; FVC: forced vital capacity; FEV1: forced expiratory volume in first second; FEV1/FVC: forced expiratory volume in first second/forced vital capacity.

**Table 4:** Comparison of changes in serum inflammatory indexes between the two groups ($\bar{x}\pm s$).

Group	WBC (×10^9^/L)		CRP (mg/L)		IL-6 (pg/mL)	
	Before the treatment	After treatment	Before the treatment	After treatment	Before the treatment	After treatment
Group A (*n* = 33)	11.07 ± 2.28	6.42 ± 1.54^∗^	21.33 ± 7.38	5.80 ± 1.36^∗^	180.27 ± 30.05	89.62 ± 17.58^∗^
Group B (*n* = 32)	11.78 ± 3.21	8.26 ± 1.66^∗^	23.54 ± 6.89	10.11 ± 3.08^∗^	180.80 ± 34.47	102.03 ± 14.19^∗^
*t*	-1.034	-4.623	-1.247	-7.332	-0.066	-3.126
*P*	0.305	<0.001	0.217	<0.001	0.947	0.003

Note: vs. before treatment, ^∗^*P* < 0.05; WBC = white blood cell count; CRP = C-reactive protein; IL-6 = interleukin-6.

**Table 5:** Comparison of cortisol function-related indicators between the two groups ($\bar{x}\pm s$).

Group	COR (nmol/L)		ACTH (pg/mL)	
	Before the treatment	After treatment	Before the treatment	After treatment
Group A (*n* = 33)	435.15 ± 56.59	175.43 ± 39.39^∗^	64.60 ± 7.93	39.62 ± 6.54^∗^
Group B (*n* = 32)	437.93 ± 45.31	203.36 ± 40.19^∗^	63.25 ± 9.65	44.12 ± 8.95^∗^
*t*	-0.218	-2.830	0.617	-2.318
*P*	0.828	0.006	0.539	0.024

Note: vs. before treatment, ^∗^*P* < 0.05; COR = cortisol; ACTH = adrenocorticotrophic hormone.

## Data Availability

The data used to support the findings of this study are available from the corresponding author (Dr. Cheng) upon request.

## References

[1] Labaki W. W., Rosenberg S. R. (2020). Chronic obstructive pulmonary disease. *Annals of Internal Medicine*.

[2] Balkissoon R., Journal Club—COPD2020 Update (2019). Global Initiative for Chronic Obstructive Lung Disease 2020 Report and the journal of the COPD foundation special edition, moving to a new definition for COPD: "COPDGene 2019". *Chronic Obstructive Pulmonary Disease*.

[3] Duffy S. P., Criner G. J. (2019). Chronic obstructive pulmonary disease: evaluation and management. *Medical Clinics of North America*.

[4] Gloeckl R., Schneeberger T., Jarosch I., Kenn K. (2018). Pulmonary rehabilitation and exercise training in chronic obstructive pulmonary disease. *Deutsches Ärzteblatt International*.

[5] Wouters E. F., Posthuma R., Koopman M. (2020). An update on pulmonary rehabilitation techniques for patients with chronic obstructive pulmonary disease. *Respiratory Medicine*.

[6] Prieur G., Combret Y., Medrinal C. (2020). High flow nasal therapy during early pulmonary rehabilitation in patients with acute severe exacerbation of COPD: beneficial or illusory?. *Respiratory Research*.

[7] Wei P., Li Y., Wu L. (2021). Serum cortisol levels and adrenal gland size in patients with chronic obstructive pulmonary disease. *Translational Research*.

[8] Tung L. F., Shen S. Y., Chen Y. T., Shih H. H., Yan J. D., Ho S. C. (2020). Early pulmonary rehabilitation increases 6MWD and reduces CRP in hospitalized patients with severe AECOPD. *ERS International Congress 2020 Abstracts*.

[9] Ta C., Mülazimoğlu D. D., Doğan D., Öcal N., Arslan Y. (2021). Effect of pulmonary rehabilitation on patients with severe and very severe COPD and emphysema. *Medical Journal of Bakirkoy*.

[10] Riley C. M., Sciurba F. C. (2019). Diagnosis and outpatient management of chronic obstructive pulmonary disease. *JAMA*.

[11] Jerng J. S., Tang C. H., Cheng R. W., Wang M. Y. H., Hung K. Y. (2019). Healthcare utilization,medical costs and mortality associated with malnutrition in patients with chronic obstructive pulmonary disease: a matched cohort study. *Current Medical Research and Opinion*.

[12] Jie X., Xudong W., Zhihai L. (2021). AECOPD research in the past ten years: a bibliographic analysis based on Web of Science. *Annals of Palliative Medicine*.

[13] Mathioudakis A. G., Janssens W., Sivapalan P. (2020). Acute exacerbations of chronic obstructive pulmonary disease: in search of diagnostic biomarkers and treatable traits. *Thorax*.

[14] Goktalay T., Akdemir S. E., Alpaydin A. O., Coskun A. S., Celik P., Yorgancioglu A. (2013). Does high-frequency chest wall oscillation therapy have any impact on the infective exacerbations of chronic obstructive pulmonary disease? A randomized controlled single-blind study. *Clinical Rehabilitation*.

[15] Lanza F. C., Alves C. S., dos Santos R. L., de Camargo A. A., Dal Corso S. (2015). Expiratory reserve volume during slow expiration with glottis opened in infralateral decubitus position (ELTGOL) in chronic pulmonary disease: technique description and reproducibility. *Respiratory Care*.

[16] Nicolini A., Grecchi B., Ferrari-Bravo M., Barlascini C. (2018). Safety and effectiveness of the high-frequency chest wall oscillation vs intrapulmonary percussive ventilation in patients with severe COPD. *International Journal of Chronic Obstructive Pulmonary Disease*.

[17] Liu T., Kang Y., Xu Z., Lyu Y., Jia L., Gao Y. (2014). A study of the value of high frequency chest wall oscillation in patients with acute exacerbation of chronic obstructive pulmonary disease. *Zhonghua Jie He He Hu Xi Za Zhi*.

[18] Esquinas A. M., Patel B., Pravinkumar E. (2014). High-frequency chest wall oscillation in infective exacerbation of COPD: is airway secretion clearance the cornerstone?. *Clinical Rehabilitation*.

[19] Alvarenga G. D., Gamba H. R., Hellman L. E., Ferrari V. G., de Macedo R. M. (2016). Physiotherapy intervention during level I of pulmonary rehabilitation on chronic obstructive pulmonary disease: a systematic review. *The Open Respiratory Medicine Journal*.

[20] Allam N. M., Badawy M. M. (2021). Does high-frequency chest wall oscillation have an impact on improving pulmonary function in patients with smoke inhalation injury?. *Journal of Burn Care & Research*.

[21] Chakravorty I., Chahal K., Austin G. (2011). A pilot study of the impact of high -frequency chest wall oscillation in chronic obstructive pulmonary disease patients with mucus hypersecretion. *International Journal of Chronic Obstructive Pulmonary Disease*.

[22] Chuang M. L., Chou Y. L., Lee C. Y., Huang S. F. (2017). Instantaneous responses to high-frequency chest wall oscillation in patients with acute pneumonic respiratory failure receiving mechanical ventilation. *Medicine*.

[23] Halpin D., Criner G. J., Papi A. (2021). Global initiative for the diagnosis, management, and prevention of chronic obstructive lung Disease. the 2020 GOLD science committee report on COVID-19 and Chronic Obstructive Pulmonary Disease. *American Journal of Respiratory and Critical Care Medicine*.

[24] Macleod M., Papi A., Contoli M. (2021). Chronic obstructive pulmonary disease exacerbation fundamentals: diagnosis, treatment, prevention and disease impact. *Respirology*.

[25] Mbchb A., Wedzicha J. A. (2020). Definition, causes, pathogenesis, and consequences of chronic obstructive pulmonary disease exacerbations. *Clinics in Chest Medicine*.

[26] Glenk L. M., Kothgassner O. D., Felnhofer A. (2020). Salivary cortisol responses to acute stress vary between allergic and healthy individuals: the role of plasma oxytocin, emotion regulation strategies, reported stress and anxiety. *Stress*.

[27] Riek A., Schrader L., Zerbe F., Petow S. (2019). Comparison of cortisol concentrations in plasma and saliva in dairy cattle following ACTH stimulation. *The Journal of Dairy Research*.

[28] Yang F., Liu N., Hu J. Y. (2020). Pulmonary rehabilitation guidelines in the principle of 4S for patients infected with 2019 novel coronavirus (2019-nCoV). *Zhonghua jie he he hu xi za zhi = Zhonghua jiehe he huxi zazhi = Chinese Journal of Tuberculosis And Respiratory Diseases*.

[29] Liu L. Y., Zeng M., Xie C. M. (2008). Oxidative stress status in patients with chronic obstructive pulmonary disease and its relation to glucocorticoid receptor levels. *Nan Fang Yi Ke Da Xue Xue Bao*.

[30] Su L., Qiao Y., Luo J. (2022). Characteristics of the sputum microbiome in COPD exacerbations and correlations between clinical indices. *Journal of Translational Medicine*.

